The article "The Research of Maneuverability Modeling and Environmental Monitoring Based on a Robotic Dolphin" was published in 2021. Journal: Appl Bionics Biomech.

# The Research of Maneuverability Modeling and Environmental Monitoring Based on a Robotic Dolphin

**DOI:** 10.1155/2021/4203914

**Published:** 2021-12-28

**Authors:** Zhibin Xue, Liangliang Li, Yixiao Song

**Affiliations:** ^1^College of Chemical Engineering, Qinghai University, Xining 810016, China; ^2^College of Mechanical Engineering, Qinghai University, Xining 810016, China; ^3^Shandong Labor Vocational and Technical College, Jinan 250022, China

## Abstract

In this study, the C-turning, pitching, and flapping propulsion of a robotic dolphin during locomotion were explored. Considering the swimming action required of a three-dimensional (3D) robotic dolphin in the ocean, we propose a maneuverability model that can be applied to the flapping motion to provide precise and stable movements and function as the driving role in locomotion. Additionally, an added tail joint allows for the turning movement with efficient parameters obtained by a fluid-structure coupling method. To obtain a mathematical model, several disturbance signals were considered, including systematic uncertainties of the parameters, the perpetually changing environment, the interference from obstacles with effective fuzzy rules, and a sliding mode of control. Furthermore, a combined strategy of environment recognition was used for the positional control of the robotic dolphin, incorporating sonar, path planning with an artificial potential field, and trajectory tracking. The simulation results show satisfactory performance of the 3D robotic dolphin with respect to flexible movement and trajectory tracking under the observed interference factors.

## 1. Introduction

Due to considerable scientific advancement in recent years, underwater robots have transformed from abstract models to more advanced prototypes, and they have been widely used in a variety of fields, including agricultural fishing, groundwater resource detection, military affairs, and environmental protection. As underwater robots have become more integrated in these fields, the motion performance of the robots has still been somewhat restricted, particularly with respect to high propulsive efficiency and flexible maneuvering.

Due to the continuous efforts of scholars, underwater robots have transformed from abstract models to prototype ones, and they have been widely used in various fields, such as fishing grounds, groundwater resources detection, military affairs, and environmental protection. As the integration level of underwater robots for various tasks has increased, their motion performance has been restricted to varying degrees, especially in terms of high propulsive efficiency and flexible maneuvering.

To demonstrate the excellent propulsion performance of fish in water, researchers have developed and launched a variety of applications to explore underwater robots that use fish-like propulsion mechanisms. Because of the pressures of natural selection, fish are shaped to have excellent propulsion parameters that help them adapt to environmental changes. To a large extent, the advantages of fish have promoted the development of underwater robots, and Tong et al.'s [1] research work focused on finding a substitute for the propeller. To achieve excellent propulsion, Scaradozzi et al. [2] used a fluid mechanics method to analyze the characteristics of BCF (body and/or caudal fin) swimming. This idea has attracted a large number of scholars worldwide, e.g., the research on tuna by Chen et al. [3]. Nguyen et al. [4] explained the dynamic modeling of the caudal fin model, and Liu and Hu [5] used a new method of oscillating wave approximation to study the advancement of robotic fish. Wang and Tan [6] studied the development of the mechanical structure of robotic fish, while Wang et al. [7] examined their propulsion using a drag coefficient. Vo et al. [8] studied the coefficient of propulsion of robotic fish with towing; and Wang et al. [9] optimized a control strategy to study the advancement of robotic fish. Further, researchers have drawn upon the advantages of dolphins to improve the performance of underwater robots. Although Ren et al. [10] and Rui et al. [11] were the first to apply this idea, they used an inaccurate method for stress analysis. Therefore, the mechanical structure of robotic fish was refined using the force analysis and research process. For example, the friction force and pressure difference are broken down into two different forces while considering the interaction between solid and fluid. Liu et al. [12], Wu et al. [13, 14], and Yuan et al. [15] performed significant work in controlling; however, they did not consider the interactions with the environment.

Many researchers have explored the manipulation characteristics and advantages of swimming mechanisms of fish. Suebsaiprom et al. [16] studied the multimodal motion of robots, and Ren et al. [17] investigated the acute turning of a robotic fish. Bal et al. [18] developed a multitask control theory for robotic fish, while Yang et al. [19] used fault-tolerance analysis methods to study operability when the robotic fish had trouble swimming. Ren et al. [20] used a data-driven method to explore operation performance, and Suebsaiprom et al. [21] studied the swimming and turning behaviors of robotic fish under the disturbance of ocean currents. Wu et al. [22] investigated forward and backward swimming to study the mobility of robotic fish; Wu et al. [23] realized the 3D movement of a robotic fish, and Xie et al. [24] studied multimodal motion control. However, despite this wealth of research on underwater robots generally, there is a lack of research on how to implement the propulsion of robotic fish by means of a flapping motion. In this study, a motion model that can effectively simulate the movement of dolphins was established. The machine dolphin was used to build dynamic models of flapping motion, pitching motion, and turning motion. Next, the fuzzy sliding mode control (SMC) strategy was adopted to carry out propulsion performance control and path tracking on the machine dolphins. During the path tracking process, the necessary interference signals and obstacles were implanted. Our results demonstrate that the robot that simulates a dolphin's movements can achieve good maneuverability and propulsion performance.

Many researchers have studied to achieve efficient propulsion performance [25–27]. However, they conducted research on two-dimensional (2D) planes or used simple geometry in 3D space. Zhang et al. [28] used the fluid-structure (F-S) coupling method to study the relationship between frequency swing and swimming based on the wing model. Chung et al. [29] used the same method to study the relationship between frequency swing and structural displacement based on thin-walled parts. Ghaffari et al. [30] proposed an interaction simulation algorithm based on a 2D wing model and verified the effectiveness of the algorithm through the F-S coupling method. Zhou et al. [31] studied the near-body pressure distribution of robotic fish using a wing model and F-S coupling method. Li et al. [32] used the CFD method to study the lift and drag coefficients of a glider. Tang et al. [33] studied the impact of population migration on the surrounding environment based on elliptical fish. Bergmann et al. [34] investigated the propulsion performance from the perspective of fluid feedback affecting the fish body based on a 2D aircraft wing. Xia et al. [35] studied the head flapping of a 3D robotic fish. However, the F-S coupling method was rarely used to optimize the motion parameters of joints based on 3D robotic fish. To solve the two-link rigid-flexible wing control problem, a boundary control approach was proposed by He et al., which was inspired by the principle of bionics to improve the mobility and the flexibility [36]. Virgala et al. developed a snake robot for planar motion in pipes. The mathematical model of the developed robot was proposed to analyze the influence of input parameters. The simulations and experiments were presented to validate the effectiveness of the proposed method and prototype [37].

This paper proposes a robotic fish that simulates dolphins in a robotic space. Dynamic simulations and the F-S coupling method were used to optimize the joint motion parameters to obtain efficient propulsion performance. Based on the optimization results, a simulated verification of the propulsion performance was conducted based on the machine dolphin.

## 2. Design of Structural Model

The speed and torque of the motor were transmitted to a pair of gears through the coupling, shaft, and key, and the crankshaft was rotated periodically. Therefore, the slider was set to move linearly on the guide bar in a reciprocating manner. The gear drove the gear to rotate through a rack fixed on the moving slider to adapt to this relationship. The tail link could achieve a certain flapping angle through the coupling, shaft, and key. The other motor was fixed on the first joint to realize the flapping motion. The output shaft and bevel gear shaft were mechanically fixed by sleeve coupling, which rotated the shaft fixed with another bevel gear periodically. Therefore, the tail link was driven up and down and fixed on the shaft. The caudal fin was divided into two halves. The bolt was mechanically connected to the tail link. Thus, a complete flapping wing mechanism model was developed.  Figure 1 shows a three-ontology model, and Figure 2 presents a simplified geometric model.

### 2.1. Dynamic Modeling of Swimming

The flapping motion is a common pattern in nature. It is a motion, which helps dolphins swim in a straight line for a long period of time and shows the higher propulsion efficiency of machine dolphins. According to the designed 3D structure model of the machine dolphin, when it is in this motion state, the first joint of its tail, pectoral fin, and dorsal fin do not move; hence, the machine dolphin can be regarded as an open-loop linear rigid body component system. As shown in Figure 3, the *X*_0_‐*Y*_0_‐*Z*_0_ coordinate system is the world coordinate system that is fixed on Earth. The positive direction of *X*_0_ is the direction in which the machine dolphin swims forward, the positive direction of *Y*_0_ is the direction in which the dolphin tail fin flaps and rises, and the positive direction of *Z*_0_ is determined according to the right-hand spiral rule. The *X*_1_‐*Y*_1_‐*Z*_1_ coordinate system is fixed at the front end of the machine dolphin, and the positive direction of each coordinate axis is consistent with the positive direction of the corresponding coordinate axes of the world coordinate system. The original center of the *X*_2_‐*Y*_2_‐*Z*_2_ coordinate system coincides with the center of mass of the head part. The positive direction of *X*_2_ indicates the swimming direction of the machine dolphin along the simplified head rod, and the positive direction of *Y*_2_ is the vertical head to the machine. The dolphin's tail fin flaps in the rising direction, and the positive direction of *Z*_2_ is determined according to the right-hand spiral rule. The original centers of the *X*_3_‐*Y*_3_‐*Z*_3_, *X*_4_‐*Y*_4_‐*Z*_4_, and *X*_5_‐*Y*_5_‐*Z*_5_ coordinate systems coincide with the center of mass of their parts. The forward direction of each coordinate axis is set according to the forward determination method of the *X*_2_‐*Y*_2_‐*Z*_2_ coordinate system; *r*^1^_0_ is the position vector of *X*_1_‐*Y*_1_‐*Z*_1_ in the coordinate system *X*_0_‐*Y*_0_‐*Z*_0_, and *r*^*i*^_0_ is the position vector of the *i*^th^ joint centroid in the coordinate system *X*_0_‐*Y*_0_‐*Z*_0_. Further, *r*^*i*^_1_ is the position vector of the *i*^th^ joint centroid in the coordinate system *X*_1_‐*Y*_1_‐*Z*_1_. *L*_2_, *L*_3_, *L*_4_, and *L*_5_ are the lengths of the head, turning joint, tail second joint, and tail third joint, respectively, *Ф*_4_ is the included angle between the second joint of the tail and the turning joins, and *Ф*_5_ is the included angle between the third joint of the tail and the second joint of the tail.

(1) $$\begin{array}{c} r_{ig}=r_{i}^{0}=r_{1}^{0}-T_{i}^{0}r_{i}^{1}, \end{array}$$

(2) $$\begin{array}{c} \omega_{ig}=\omega_{i}^{0}=\omega_{1}^{0}-{T_{\theta }}_{i}^{0}Y_{i}^{0}, \end{array}$$

(3) $$\begin{array}{c} \nu_{ig}=\nu_{i}^{0}=\nu_{1}^{0}-\omega_{i}^{0}\times r_{i}^{0}, \end{array}$$

(4) $$\begin{array}{c} \alpha_{ig}=\alpha_{i}^{0}=\omega_{i}^{1}+\omega_{1}^{0}\times \omega_{i}^{0}, \end{array}$$

(5) $$\begin{array}{c} a_{ig}=a_{i}^{0}=\nu_{i}^{1}+\omega_{1}^{0}\times \nu_{i}^{0}. \end{array}$$

For the analysis and simplification of the model, the geometry was simplified according to the robot's flapping principle. The head of the dolphin always moves horizontally; hence, the first joint of the tail of the object with the head as the reference was connected to the tail link in the same way through a movable hinge.

#### 2.1.1. Dynamic Modeling of the Third Joint of the Tail

During the up and down flapping motion, the second joint of the machine dolphin tail fin connecting rod was shorter than the machine dolphin flapping movement; and the 3D body design rigidly connected the tail fin and the tail fin connecting rod. Because of the effect of rod motion synchronization, the caudal fin link and caudal fin were regarded as components in the geometrically simplified model. Therefore, the mechanical dolphin caudal fin and caudal fin link were regarded as joints for the dynamic analysis. However, considering that the shell corresponding to the caudal fin connecting rod was relatively large, the shell external force was equivalent to the position of the center of mass of the second joint of the machine dolphin flapping motion, thereby generating an equivalent combined external force and an equivalent moment of force. The combined external force and moment of the first joint of the machine dolphin flapping motion were combined and processed. The tail fin of the dolphin was a thin-walled piece, and its thickness was much smaller than the length and width of the tail fin. Therefore, the tail fin was regarded as a 2D flat plate, and a force analysis was performed. According to the 2D plate theory of robot fish established by Chopra [38], the force of the fluid on the thin-walled member in the thickness direction was far less than the positive pressure and shape resistance. Thus, the flow velocity of the fluid in the thickness direction was negligible. As shown in Figure 4, to simplify the fluid environment, the fluid velocity is always kept constant and the wind environment does not affect it. Equations (6)–(10) describe the model parameters. The hydrodynamic coefficients, like lift coefficient, pressure coefficient, drag resistance coefficient, friction coefficient, and other coefficient, are obtained via computational fluid dynamics (CFD) simulation.

(6) $$\begin{array}{c} F_{5s}=2\pi \rho C_{s}A_{5}{\upsilon_{5}}^{2}\sin\sigma_{5}, \end{array}$$

(7) $$\begin{array}{c} F_{5s}=2\pi \rho C_{s}A_{5}{\upsilon_{5}}^{2}\sin\sigma_{5}, \end{array}$$

(8) $$\begin{array}{c} F_{5p}=c_{p}\left[0.5\rho \left(\upsilon_{5}^{2}-\upsilon_{s}^{2}\right)-\rho \frac{\partial \sigma_{5}}{\partial t}\right], \end{array}$$

(9) $$\begin{array}{c} F_{5d}=\pi \rho A_{5}c_{d}^{2}\left(\frac{d\upsilon_{5}}{dt}\cos\delta_{5}+\frac{d\cos\delta_{5}}{dt}\upsilon_{5}\right), \end{array}$$

(10) $$\begin{array}{c} F_{5u}=2\pi \rho C_{s}A_{5}{\upsilon_{5}}^{2}\cos\left(\sigma_{5}-\delta_{U}\right), \end{array}$$

where *c*_*s*_ = 1040sin(8*t*/*t*_max_ + 1.5), *c*_*n*_ = *μυ*_5_*L*_3_, *c*_*d*_ = 16.99*FR*∗Re^0.47^, *c*_*f*_ = 0.8, and *c*_*v*_ = 0.64(Θ_5_/*υ*_*s*_) − 0.5. *F*_5_ is the lift of the tail fin, *F*_5*p*_ is the pressure resistance of the effective longitudinal surface of the caudal fin, *F*_5*m*_ is friction, *F*_5*d*_ is the drag, and *F*_5*u*_ is the induced resistance. *A*_5_ is the surface area of the tail fin, *c*_*s*_ is the lift coefficient, *c*_*p*_ is the pressure coefficient, *c*_*d*_ is the drag resistance coefficient, *c*_*f*_ is the coefficient of friction, *c*_*n*_ is the coefficient of the dynamic viscosity, *c*_*v*_ is the longitudinal coefficient of the frictional resistance, Θ is the surface temperature of the machine dolphin, and Re is the Reynolds number. In Equation (11) [22], *F*^∗^_5*g*_ is the inertial force of the inertial caudal fin, *M*^∗^_5*g*_ is the inertial moment of the caudal fin, and *I*_5_ is the rotational inertia of the caudal fin.

(11) $$\begin{array}{c} \left[\begin{array}{c} F_{5g}^{*}\\ M_{5g}^{*} \end{array}\right]=-I_{5}\left[\begin{array}{c} a_{5}\\ a_{d} \end{array}\right]+I_{5}\left[\begin{array}{c} \omega_{5}\times \upsilon_{5}\\ \omega_{5}\times \omega_{5} \end{array}\right]. \end{array}$$

#### 2.1.2. Dynamic Modeling of the Second Joint of the Tail

The force on the connecting rod housing was equivalently replaced by the combined force and external moment acting on the center of mass. However, such housing has a certain volume, which makes the theory of flat plates unusable. The middle trapezoidal interface was affected by shape resistance. A force analysis diagram of the second joint is shown in Figure 5, and Equations (12)–(18) describe the model parameters.

(12) AY4=πRm2,

(13) AX4=L3RQ+RH,

(14) Fh5x=0.5ρcxA5υ52,h5Fy=0.5ρcyA5υ52,

(15) F5f=Fh5x2+h5Fy20.5,

(16) M5f=Fh5x2+h5Fy2L2sinθ3,

(17) Fh4x=0.5ρcAX4υ42,h4Fy=0.5ρcdAY4υ42,

(18) F4u=Fh4x2+h4Fy20.5.

*R*_*Q*_ is the anterior cross-sectional radius of the second joint, and *R*_*H*_ is the posterior cross-sectional radius. _*X*_*A*_4_ is the cross-sectional area of the second joint in the horizontal intermediate layer; _*Y*_*A*_4_ is the cross-sectional area of the second joint in the vertical intermediate layer, and *R*_*m*_ is the radius of the second joint in the vertical intermediate layer. The shell of the third joint connecting rod can be regarded as a round plastic table structure. *F*_5*f*_ is the additional external force of the third joint connecting the rod shell, *M*_5*f*_ is the additional external moment of the second joint connecting the rod shell, _*X*_*A*_5_ is the area of the third joint horizontal intermediate layer section, _*Y*_*A*_5_ is the area of the second joint vertical intermediate layer section, and *F*_4*u*_ is the water resistance of the second joint. The remaining forces refer to the caudal fin modeling method. All forces are decomposed horizontally and vertically as shown in Appendix.

#### 2.1.3. Kane Modeling of Flapping

According to the above analysis of each component, the total active force, total active moment, total inertia force, total inertia moment, and moments provided by the two motors were obtained. Using Kane's dynamics equation, *K*_*PG*_ (the generalized inertial force) and *K*_*pG*_ (the generalized main power) were determined to obtain the flapping motion dynamic model, as presented below.

(19) $$\begin{array}{c} K_{PG}=\overset{2}{\underset{1}{\sum }}\left(\frac{\partial \upsilon_{i}}{\partial \overset{.}{\theta }}F_{pG}+\frac{\partial \omega_{i}}{\partial \overset{.}{\theta }}M_{pG}\right),\\ K_{PZ}=\overset{2}{\underset{1}{\sum }}\left(\frac{\partial \upsilon_{i}}{\partial \dot{q}}F_{pz}+\frac{\partial \omega_{i}}{\partial \dot{q}}M_{pz}+\frac{\partial \omega_{i}}{\partial \dot{q}}M_{pd}\right),\\ K_{PZ}+K_{PG}=0. \end{array}$$

### 2.2. Dynamic Modeling of C-Turning

Underwater robots need to search for objects, avoid obstacles, adjust yaw, and perform such other actions; all these actions depend on a high degree of maneuverability. Due to the high mobility and maneuverability of fish in the ocean, researchers have focused on creating bionic/robotic fish, seeking inspiration from natural fish for innovative design points with function with high mobility. Among these sources of inspiration, ocean dolphins are particularly inspiring, due to their ability to make complex movements, such as quick u-turns, rotations in space, dives, and pitches. Because maneuvering plays an important role in the course correction of search modes, obstacle avoidance, and external interference, the turning problem is regarded as a typical maneuvering behavior. The machine dolphin uses a pair of pectoral fins to control the turning direction and a flexible spine to bend. These two actions cooperate to achieve the turning action. Its turning speed is as high as 450° per second, and the turning radius is as low as 11–17% of the body length [39]. Su et al. proposed C-starts algorithm for a BCF-type multijoint robotic fish [40]. The faster C-starts can be achieved by concatenated multilink mechanism, such as four yaw joints. The designed robotic dolphin of this manuscript consists of two pitch joins (the second and third joints) and a yaw joint (the first joint). The propulsion can be achieved by dorsoventral oscillations through the pitch joints, and the yaw maneuver can be realized through the combination of the yaw joint and a pair of 2-DOF mechanical flippers. This is the difference between the two papers in mechanical structure. From [40], the C-start turning is defined as three stages: turn swiftly, propulsive, and steady swimming. The C-turning of this manuscript can be achieved through sharp bending, keeping, and slowly recoiling. The difficulty of controller design is reduced by adjusting only one yaw joint. This is the difference between the two papers in controllability. Pham et al. [41] used a controller to control the steering movement that relies on the pectoral and dorsal fins. Li et al. [42] studied the coordinated turning characteristics achieved with the pectoral and caudal fins. Weihs [43] observed the turning movements of various fish and obtained a turning curve. Liu et al. [44] proposed a new method for robotic fish steering movements, while Yu et al. [45] proposed a method to achieve plane steering of machine dolphins. Based on Kane's dynamics modeling method, the dynamic equations of the steering motion of the dolphin robot were established, and its effective steering motion was realized. To study the relationship between the turning radius, propulsion speed, and propulsion force, a fluid coupling analysis was carried out.

For the machine dolphin C-type rotational motion, the first joint of the machine dolphin's tail performs C-type rotation in the *X*_0_‐*O*_0_‐*Z*_0_ world coordinate system; thus, the steering gear activates the two output shafts at the position of the rotating joint, and the tail follows the first joint. The first joint of the tail of the machine dolphin swings left and right in the *X*_0_‐*O*_0_‐*Y*_0_ coordinate system; i.e., the motors of the second and third joints of the tail of the machine dolphin do not work in this motion state. *X*_1_‐*O*_1_‐*Y*_1_ is the same as *X*_2_‐*O*_2_‐*Y*_2_ and the up-and-down flapping coordinate system, *X*_6_‐*O*_6_‐*Y*_6_ and *X*_7_‐*O*_7_‐*Y*_7_ are the left and right pectoral fin centroid coordinate systems, respectively; *X*_BZ_‐*O*_BZ_‐*Y*_BZ_ is the machine dolphin centroid coordinate system, and *X*_ZZ_‐*O*_ZZ_‐*Y*_ZZ_ is the center-of-mass coordinate system of the tail part of the machine dolphin turning movement. *L*_0_ is the length of the head, and *L*_ZW_ is the length of the tail joint of the machine dolphin turning movement. The orthogonal direction vector of the coordinate axis in the steering link coordinate system series is set according to the orthogonal direction vector of the coordinate axis in the coordinate system series in the machine dolphin flap analysis, as shown in Figure 6.

(20) $$\begin{array}{c} F_{2D}=c_{c1}\nu_{z0}^{2}A_{0H}\mathrm{sign}\left(s_{*}\right),\\ F_{2c}=c_{c2}\nu_{z0}^{2}A_{zzz}\mathrm{sign}\left(s_{*}\right),\\ F_{cD}=c_{c1}\nu_{zz}^{2}A_{zzH}\mathrm{sign}\left(s_{*}\right),\\ F_{cz}=c_{c2}\nu_{zz}^{2}A_{WH}\mathrm{sign}\left(s_{*}\right),\\ F_{zn}=-F_{2c}\cos\theta_{0}+F_{2D}\sin\theta_{0}+F_{cD}\sin\theta_{0}+F_{cz}\cos\theta_{0},\\ F_{zt}=F_{2c}\sin\theta_{0}+F_{2D}\cos\theta_{0}+F_{cD}\cos\theta_{1}+F_{cz}\sin\theta_{1},\\ M_{ZB}=0.5\left(L_{0}F_{2c}+L_{zw}F_{cZ}\right),\\ \left[\begin{array}{c} F_{cg}^{*}\\ M_{cg}^{*} \end{array}\right]=-I_{cZ}\left[\begin{array}{c} a_{cg}\\ \alpha_{cw} \end{array}\right]+I_{cZ}\left[\begin{array}{c} \omega_{cg}\times \upsilon_{cZ}\\ \omega_{cg}\times \omega_{cg} \end{array}\right],\\ K_{cG}=\overset{2}{\underset{1}{\sum }}\left(\frac{\partial \upsilon_{i}}{\partial \dot{\theta }}{F^{*}}_{cg}+\frac{\partial \omega_{i}}{\partial \dot{\theta }}{M^{*}}_{cg}\right),\\ K_{cZ}=\overset{2}{\underset{1}{\sum }}\left(\frac{\partial \upsilon_{i}}{\partial \dot{\theta }}\left(F_{zn}+F_{zt}\right)+\frac{\partial \omega_{i}}{\partial \dot{\theta }}M_{ZB}\right),\\ K_{cZ}+K_{cG}=0. \end{array}$$

Here, *F*_2*D*_ and *F*_2*C*_ are the combined lateral external resistance and combined longitudinal external resistance, respectively, of the mass center of the head of the robotic dolphin, *F*_*CD*_ and *F*_*CZ*_ are the combined lateral external resistance and combined longitudinal external resistance, respectively, of the mass center of the tail of the robotic dolphin, *F*_*ZN*_ is the combined external force in the normal direction of the turning track of the robotic dolphin at a certain time, and *F*_*CT*_ is the tangent square of the turning track of the robotic dolphin at a certain time. *M*_*ZB*_ is the active closing moment of the robotic dolphin at a certain time, *f*^∗^_*CG*_ is the inertial closing moment of the robotic dolphin at a certain time, *m*^∗^_*CG*_ is the inertial closing moment of the robotic dolphin at a certain time, *U*_0_ is the relative speed of the head center of mass of the dolphin robot, *u*_*zz*_ is the speed of the turning tail center of mass of the robotic dolphin, *u*_*cz*_ is the overall relative propulsion speed of the robotic dolphin, and *a*_0*h*_ is the cross-sectional area of the head center of mass of the robotic dolphin. *A*_*zzz*_ is the longitudinal cross-sectional area of the mass center of the head of the robotic dolphin, *A*_*zzH*_ is the transverse cross-sectional area of the mass center of the turning tail fin of the robotic dolphin, *A*_*WH*_ is the longitudinal cross-sectional area of the mass center of the turning tail fin of the robotic dolphin, *C*_*c*1_ and *C*_*c*2_ are the transverse hydrodynamic coefficient and the longitudinal hydrodynamic coefficient of the robotic dolphin, *I*_*cz*_ is the overall moment of inertia when the robotic dolphin rotates, *a*_*cG*_ is the overall acceleration of the mass center of the robotic dolphin, and *α*_*cW*_ is the rotational angular acceleration of the dolphin's whole center of mass; *ω*_*cG*_ is the rotational angular velocity of the dolphin's center of mass, *K*_*cG*_ is the generalized inertial force of C-type steering, and *K*_*cZ*_ is the generalized active force of C-type steering.

Such as *L*_*i*_, *θ*_*i*_, *Ф*_*i*_, *μ*, Re, *M*, *F*, *I*, *A*, *δ*, *ρ*, Θ, *c*_*i*_, *r*_*i*_^*j*^, *ω*, *υ*, *α*, and *a*, all mathematical symbols include the meaning of each symbol in Section 2, which are as shown in Glossary.

## 3. Motion Simulation Based on ADAMS

The constraints between the tail joint and the rotation axis of the tail, intermediate joint, and rotation axis of the head were set as cylinder constraints. The constraints between the intermediate joint and the rotation axis of the tail and between the head and rotation axis of the head were set as fixed constraints. The transmission condition of the head shaft was set to 15 *d*∗sin (times). The spin drive condition was 15 *d*∗cos (times). The force sensor was placed at the center of mass of the robotic dolphin's head, and the direction of which was the tangential direction of the movement track of the center of mass of the head. Two speed sensors were placed at the center of mass of the head shaft and tail shaft. The moving time range was set to 15 s, and the number of moving steps was set to 500 steps. The analysis type was set to the dynamic mode. We chose to start in equilibrium; if it needed to be reset first when restarting, it could be run. The overall dynamic mechanism design of the robotic dolphin based on ADAMS is shown in Figure 7. The display diagrams of the flapping wing simulation environment variables and the turning simulation environment variables are shown in Figure 8(a). Figures 8(b)–8(d) are the components of the two axis moments in the flapping motion and the head force in the *Y* and *Z* directions in the rotational motion, respectively.

## 4. Performance Optimization with Fluid-Structure (F-S) Coupling

### 4.1. Performance Optimization about Flapping

In this study, we used F-S coupling to optimize joint motion parameters, as shown in Figure 8 and Tables 1–3. When the robotic dolphin is swimming, it is affected by the resistance in front of it. Therefore, the flow direction of the outflow field should prevent the dolphin robot from moving forward. The inlet flow rate was set to 20 m/s, and the outlet pressure was set to 0 Pa. The joint beat frequency, maximum amplitude, and phase difference were the same as those in ADAMS. The joint tapping frequency, maximum tapping amplitude, and joint phase difference as a function of propulsion speed and propulsion force were constraints for the optimization of the overall joint motion parameters, as shown in Tables 1–3.

The relationship between each parameter and propulsion effect is obtained by the fluid-solid coupling method; but the influence of each parameter on the motion of the entire joint and the propulsion effect need to be optimized. Therefore, the APSO is used to optimize the overall propulsion effect. The APSO optimization algorithm is a swarm intelligence optimization algorithm [46], and it is described in Procedure 1. The objective function is set to the maximum power, as shown in Equation (21). The constraints are presented in Table 4, and the optimization results are presented in Table 5.

(21) $$\begin{array}{c} \mathrm{MAX}{\left({\left(F_{4t}u_{4}\right)}^{2}+{\left(F_{5t}u_{5}\right)}^{2}\right)}^{0.5}. \end{array}$$

### 4.2. Performance Optimization of C-Turning

For steering movement, the C-steering movement is an index to measure the athletic ability of the robotic dolphin. The results of this robot-based F-S coupling method to study the influencing factors of the turning radius are shown in Figure 9.

(22) $$\begin{array}{c} F_{cn}=m_{bd}\omega_{cz}^{2}r_{cz},\\ \omega_{cz}=163.26{\left(\frac{r_{cz}}{L_{BD}}\right)}^{-0.66}, \end{array}$$

where *m*_*bd*_ is the sum of the overall mass and the additional mass of the robotic dolphin, *r*_*cz*_ is the turning radius of the robotic dolphin at a certain time, *ω*_*cz*_ is the turning angular speed of the robotic dolphin at a certain time, and *L*_*BD*_ is the overall length of the robotic dolphin. The results of optimization effect on turning radius are shown in Figure 10.

## 5. Overall Control Strategy

In the motion control strategy module, methods such as environment detection, obstacle avoidance, and path tracking are used for the design. The sonar head was used for environment detection, the artificial potential field (APF) method was used for obstacle avoidance, and the fuzzy sliding mode controller was used for path tracking, as shown in Figure 11. Yang et al. [47] used a sliding mode observer to observe motor torque.

### 5.1. Environmental Monitoring with Sonar

The working environment of dolphins is a complex and dynamic natural environment. Therefore, obstacles that may appear during actual movement must be considered. To avoid obstacles, a sensor must be used to detect the distance of the objects. The safe area in the process of avoiding obstacles was calibrated according to the detection distance and the reverse direction. One of the main characteristics of dolphins and their obstacle avoidance strategies is their use of sound. The sonar used in the present study was designed using the sound of the robotic dolphins. This is similar to previous work conducted by Wang et al. [48], who controlled an underwater robot in a predicted situation using sonar.

This study used a multisensor strategy to identify the swimming environment of dolphins. Three sonar sensors presented the working environment of the machine dolphins and uploaded it to the host computer wirelessly. One was placed in front of the detection environment, and the other two were placed on the left and right sides of the dolphins of the detection machine. The positions of the three sonar sensors on the integrated control board of the head of the dolphin robot are shown in Figure 12(a). Figures 12(b)–12(d) show an example of environmental monitoring with a sonar for measuring the depth of the underwater mine.

### 5.2. Obstacle Avoidance Design

There are many algorithms for obstacle avoidance; in this study, an APF algorithm was used. The obstacle avoidance principle adopts the principle of near repulsion and far absorption. When the robotic dolphin is repelled on the external force table or when the external potential of the safety zone is set, the dolphin robot attracts the external force, as described in

(23) $$\begin{array}{c} {\dot{x}}^{i}=-\nabla_{x^{i}}\delta \left(x^{i}\right)+\underset{j=1,j\neq i}{\sum }g\left(x^{i}-x^{j}\right),\;i=1,\cdots ,M, \end{array}$$

where *x*^*i*^ ∈ *R*_*n*_ represents the position of individual *i*, −∇_*x*^*i*^_*δ*(*x*^*i*^) stands for the collective motion's direction resting with the different social attractant/repellent potential field environment profile around individual *i*, and *g*(.) represents the function of attraction and repulsion between the individual members.

Figure 13 shows the isotropic swarm foraging behavior control simulation, in which the social swarms in a multiobstacle environment are tracked. The vertical and horizontal coordinates in Figure 13 represent the position coordinates in the plane, and their units are in m; “∗” represents the starting point of multiple robotic dolphins, the black circles represent obstacles, the red circle represents the target point, and green represents the walking path of the robotic dolphins.

### 5.3. Path Planning and Trajectory Tracking

In this study, the fuzzy SMC strategy was used to control the path tracking of the robotic dolphin. Kelasidi et al. [49] studied a path following a line by using a physical USR. Chen et al. [46] studied the effect of path tracking using the line-of-sight method combined with the fuzzy control strategy and a genetic algorithm.  Table 6 lists the fuzzy rules for promoting efficacy. Suebsaiprom et al. [21] used an SMC strategy to track 2D and 3D paths during the development of a slender vehicle. However, in that study, they did not use a real environment and therefore provided no solutions for interference signals and obstacles. Xu et al. [50], alternatively, designed an anti-Gaussian disturbance program with random variables for tracking the paths for unmanned aerial vehicles (UAVs). Based on this prior research, an SMC scheme was adopted in the present study, incorporating the advantages of the sliding mode. Li et al. [51] used SMC for path tracking for a tracked robot that can operate in soft and sticky soil. Das et al. [52] used the Q-learning method to find an effective method in a complex environment, which verified the excellent performance of APF in path planning. Ma et al. [53, 54] optimized the sliding mode system, and Xue et al. [55] used the MRRT∗-connect algorithm for the path planning of the USV. Therefore, the rapid and effective path planning strategies in the above references for the robotic dolphin provide a solid basis for underwater swimming. Bozek et al. developed a path planning algorithm for the control of a wheeled robot. Two artificial neural networks were utilized to ensure steering optimal motion. The results confirmed the efficiency of the proposed control algorithm for the mobile robot to move to the point with a given position and a given orientation [56]. He et al. [57] investigated the trajectory tracking problem of flapping-wing micro aerial vehicles. An adaptive control scheme is proposed, which included the saturated position controller, attitude controller, and a radial basis function neural network. Simulations are carried out to verify the effectiveness of the proposed control scheme.

#### 5.3.1. Design of Sliding Mode Controller

Nonlinear and incomplete system control can be realized according to the sliding mode. The SMC method is used to control the position and attitude of the robotic dolphin and track it with a straight line and curve. However, there are many uncertain coefficient parameters in the dynamic modeling of a dolphin robot. This makes the SMC unable to control the robotic dolphin effectively. Therefore, this study adopts the method of generating fuzzy rules through combining fuzzy and sliding modes, which can effectively track the trajectory.

(24) η˙tr=RGBUtr,

(25) η¨tr=R˙GBUtr+U˙trRGB,

(26) U˙tr=R˙GBη˙tr+RGBη¨tr,

where *η*_*tr*_ is the generalized position in the plane of motion of the robot dolphin, *U*_*tr*_ is the velocity vector in the plane of motion of the robotic dolphin, and ^*G*^*R*_*B*_ is the transformation matrix mapped from the fixed coordinate system in the plane of motion of the robotic dolphin to the world coordinate system.

(27) $$\begin{array}{c} M\left(U_{tr}\right){\dot{U}}_{tr}+N\left(U_{tr}\right)=\tau_{U_{tr}}^{tr}, \end{array}$$

where *M*(*U*_*tr*_) is the composite matrix of the mass of the dolphin, including the mass and additional mass of the dolphin model. *N*(*U*_*tr*_) is the superposition matrix of Coriolis, centripetal term, and damping matrix of the dolphin, the composite matrix of the generalized external force, the generalized moment of the dolphin, and the superposition matrix of the external interference force. By substituting Equations (24)–(26) into (27), we obtain

(28) $$\begin{array}{c} M\left(\eta_{tr}\right){\ddot{\eta }}_{tr}+N\left(\eta_{tr},{\dot{\eta }}_{tr}\right)=\tau_{U_{tr}}^{tr}. \end{array}$$

To effectively realize the sliding mode tracking system control based on the pose state of the robotic dolphin, the control error of its position motion in the world coordinate system and the change error of the combination matrix of the linear velocity and the angular velocity of the robot dolphin in the fixed coordinate system are formulated, as shown below.

(29) $$\begin{array}{c} \left\{\begin{array}{c} e_{1}=\eta_{tr}-\eta_{dtr},\\ e_{2}=U_{tr}-U_{dtr}. \end{array}\right. \end{array}$$

For plane motion tracking of the robotic dolphin, the first-order sliding surface is used here, as in

(30) $$\begin{array}{c} s_{tr}=c_{c}e_{1}+e_{2}, \end{array}$$

(31) $$\begin{array}{c} \dot{s}=c_{c}{\dot{e}}_{1}+{\dot{e}}_{2}=-M^{-1}\left(\eta_{tr}\right)N\left(\eta_{tr},{\dot{\eta }}_{tr}\right)+M^{-1}\left(\eta_{tr}\right)\tau_{\eta_{tr}}^{tr}-{\ddot{\eta }}_{tr}. \end{array}$$

To eliminate the discontinuity of the robotic dolphin affected by the external environment, the method is used to deal with the generalized external force superposition matrix by rejecting interference discontinuity.

(32) $$\begin{array}{c} \tau_{\eta_{e}}^{tr}=-\tau_{\eta_{tr}}^{tr}\left[\begin{array}{ccc} 1 & 0 & 0\\ 0 & 1 & 0\\ 0 & 0 & 1 \end{array}\right]\mathrm{sign}\left(s_{*}\right). \end{array}$$

Furthermore, the Lyapunov function is used to design the stability of the plane-motion tracking system.

(33) $$\begin{array}{c} v_{tr}=0.5{s_{tr}}^{2}\tau_{\eta_{c}}^{tr}=-\tau_{\eta_{tr}}^{tr}\left[\begin{array}{ccc} 1 & 0 & 0\\ 0 & 1 & 0\\ 0 & 0 & 1 \end{array}\right]\mathrm{sign}\left(s_{*}\right). \end{array}$$

After taking the derivative, we obtain the following

(34) $$\begin{array}{c} \dot{v}=s_{tr}\left(-M^{-1}\left(\eta_{tr}\right)N\left(\eta_{tr},\left({\dot{\eta }}_{tr}\right)\right)+M^{-1}\left(\eta_{tr}\right)\tau_{tr}-{\ddot{\eta }}_{tr}\right)\leq s\left(-\left\|M^{-1}\left(\eta_{tr}\right)\right\|\left\|N\left(\eta_{tr},{\dot{\eta }}_{tr}\right)\right\|-\left\|M^{-1}\left(\eta_{tr}\right)\right\|\tau_{\eta_{tr}}^{tr}\left\|\left[\begin{array}{ccc} 1 & 0 & 0\\ 0 & 1 & 0\\ 0 & 0 & 1 \end{array}\right]\right\|\mathrm{sign}\left(s_{tr}\right)-\left\|{\ddot{\eta }}_{tr}\right\|\right)\leq -\left\|s\right\|\sigma_{s}≺0. \end{array}$$

According to the Lyapunov function, it can be determined that the plane motion tracking control system of the robotic dolphin inevitably appears on the sliding surface, which is achieved in a limited time. The Simulink of the SMC of the robotic dolphin is shown in Figure 14.

Such as *S*, *e*, *v*, *σ*_*s*_, and *U*_*t*_, all mathematical symbols include the meaning of each symbol in Section 5.3.1, which are as shown in Glossary.

#### 5.3.2. Path Tracking in Plane

In the actual path tracking module, path switching occurs; hence, this study uses a straight line followed by a circle to have the straight path and circular path intersect at the same time, so as to investigate the problem of path switching. For the actual plane path in *m*, the simulation time was too long for the simulation. Therefore, this study adopts the equal-scale strategy, in which the actual coordinate is equal to 100 : 1 instead of the simulation coordinates. For the path function extracted in this study, Equation (35) is used. The simulation results are presented in Figure 15, in which the ideal straight-line trajectory is represented by blue solid lines, the ideal circular trajectory is represented by red solid lines, and the actual swimming path of robotic dolphins is represented by black dashed lines.

(35) $$\begin{array}{c} \left\{\begin{array}{cc} x\left(t\right)=y\left(t\right)=t, & t<1,\\ {\left(x\left(t\right)-1\right)}^{2}+{\left(y\left(t\right)-1\right)}^{2}=0.1^{2}, & t\geq 1, \end{array}\right. \end{array}$$

where *x*(*t*) and *y*(*t*) represent the *X* and *Y* coordinate points of the actual motion track of the robotic dolphin in the plane and *t* is the time variable.

Such as *x*, *y*, and *t*, all mathematical symbols include the meaning of each symbol in Equation (35), which are as shown in Glossary.

Through the simulation results, it is not difficult to conclude that when the robot dolphin goes through the straight-line path, there will be no path mutation; and the robotic dolphin will take the last point of the straight-line path as the outer point of the circular track and perform the movement of the outer point to the circular sliding surface again. The actual straight-line path tracks the direction of the last point or coincides with the actual straight-line path. When the motion direction of the robotic dolphin's starting point of the actual circular path coincides with the tangent direction of the corresponding point in the ideal circular path, the curve of the path switching process is a smooth curve; but its curvature gradually changes from zero to the curvature of the entry point of the ideal circular trajectory.

#### 5.3.3. Present Path Tracking

The actual motion belongs to the space motion of the dolphin robot. Therefore, this study attempts to track the trajectory of a dolphin robot in space. At the same time, in order to show the movement effect and effective tracking of the robotic dolphin at the starting point, two dolphins are inserted in the actual movement path to achieve the schematic effect, using Equation (36). Regular objects, such as cylinders and cuboids, replace obstacles.

(36) $$\begin{array}{c} \left\{\begin{array}{c} x\left(t\right)=\left(1+t\right)\cos t-1,\\ y\left(t\right)=\left(1+t\right)\sin t-1,\\ z\left(t\right)=0.2t. \end{array}\right. \end{array}$$

In Figure 16, it takes the horizontal plane as the reference plane and takes the entire underwater plane. It is not difficult to find that the fluctuation and error are large over a period of time after the startup. However, with the depth and time factors, the robotic dolphin tends to stabilize. The path code for the robotic dolphin's tracking is shown in Procedure 2.

## 6. Conclusions and Future Work

In this paper, a novel robotic dolphin is designed to analyze the maneuverability dynamic model, such as C-turning, pitching, and flapping propulsion. Firstly, a robotic dolphin consisting of yaw joint and two pitch joints is designed to provide the dynamic analysis platform. After that, the dynamic modeling of the robot swimming, C-turning, and dorsoventral propulsion is analyzed. Furthermore, ADAMS is used to carry out motion simulation, thereby optimizing the propulsion performance. To obtain efficient propulsion performance, the joint motion parameters of the machine dolphin are optimized using the F-S coupling method and the APSO algorithm. Finally, we propose the fuzzy sliding mode controller to realize the path tracking. In the process of tracking, sonar sensors are utilized to perceive the environment, and the APF algorithm is used to develop obstacle avoidance movements, thereby achieving autonomous path planning and tracking. To study the robustness of the control system in terms of path design, the linear path was followed by the circular path first, and path tracking autonomous switching is realized. Simulations on the robotic dolphin testify the effectiveness of the path tracking method. This work sheds light on intelligent control of robotic dolphins in 3D environments, contributing to updated design and control of innovative fish- or dolphin-inspired swimming robots.

In the future, the motion performance and 3D environmental monitoring will be systematically implemented and improved on the actual robotic dolphin platform. The practical application scenarios include water quality monitoring, fish behavior observation, and seabed salvage. Thereby, the robotic dolphin will have a better adaptability and intelligence in complex underwater environments.

## Figures and Tables

**Figure 1:** Three-dimensional distribution diagram of machine dolphin.

**Figure 2:** Equivalent model used as fluid-solid coupling.

**Figure 3:** The coordinate system of the robotic dolphin.

**Figure 4:** Force analysis of the third joint of the tail.

**Figure 5:** Force analysis of the second joint of the tail.

**Figure 6:** Diagram of dynamic analysis for C-turning. (a) Coordinate system for C-turning. (b) Force analysis for C-turning.

**Figure 7:** Diagram of motion simulation based on ADAMS. (a) Motion simulation of flapping. (b) Displacement change of turning movement. (c) Overall dynamics mechanism design of robotic dolphin based on ADAMS.

**Figure 8:** Velocity and pressure contours at the main view interface. (a) The values of frequency, amplitude, and phase are 1.5 Hz, 0.2 m, and 0 degrees, respectively. (b) The values of frequency, amplitude, and phase are 0.5 Hz, 0.2 m, and 0 degrees, respectively. (c) The values of frequency, amplitude, and phase are 1.5 Hz, 0.2 m, and 70 degrees and 0.5 Hz, 0.1 m, and 0 degrees, respectively. (d) The values of frequency, amplitude, and phase are 1.5 Hz, 0.2 m, and 20 degrees, respectively.

**Figure 9:** Results with F-S coupling for C-turning. (a) Speed chart for turning left in the *X* direction. (b) Speed chart for turning right in the *X* direction. (c) Speed chart for turning left in the *Y* direction. (d) Speed chart for turning right in the *Y* direction. (e) Speed chart for turning left in the *Z* direction. (f) Speed chart for turning right in the *Z* direction.

**Figure 10:** Optimization effect on turning radius. (a) Influence of joint rotation frequency on turning radius. (b) Influence of joint rotation angle on turning radius.

**Figure 11:** Block diagram of path tracking based on machine dolphin.

**Figure 12:** Sonar sensor detection used to identify the environment. (a) Structure diagram of sensor placement. (b) Effect diagram of sensor detection. (c) Micron DST SONAR S08725. (d) Measurement of the depth of the underwater mine.

**Figure 13:** Track of social foraging swarms in a multiobstacle environment.

**Figure 14:** Simulink of SMC of robotic dolphin.

**Figure 15:** Path tracking in plane.

**Figure 16:** Path tracking in space based on sliding mode control. (a) Trajectory tracking about curve in space. (b) Angle curve about curve in space. (c) Error curve about 3D coordinates in case of path tracking in plane in space.

**Procedure 1:** APSO.

**Procedure 2:** Path code for tracking.

**Table 1:** Influence of beat frequency.

Frequency (Hz)	0.5	1	1.5	2
Propulsion speed (10∗m/s)	1.901	3.957	3.241	1.962
Propulsion force (100∗N)	0.67363	2.46768	3.13389	1.63397

**Table 2:** Effect of maximum amplitude.

Amplitude (m)	0.1	0.2	0.3	0.4
Propulsion speed (10∗m/s)	7.594	8.06	5.104	1.491
Propulsion force (100∗N)	1.58417	4.00256	4.37939	1.68328

**Table 3:** Influence of phase difference.

Phase (degrees)	20	40	60	80
Propulsion speed (10∗m/s)	1.194	1.563	1.675	1.757
Propulsion force (100∗N)	0.63229	0.70225	0.74995	0.355948

**Table 4:** Constraint parameters.

Parameter	*f*	*ψ*	*α*	*A*_4_	*A*_5_
Range	[0, 2]	[0, pi/2]	[0, pi/12]	[0.05,0.4]	[0.05,0.4]

**Table 5:** Results of overall optimization.

Parameter	*f*	*ψ*	*A*_4_	*A*_5_
Value	1.267	1.169	0.2029	0.2589

**Table 6:** Fuzzy rules for promoting efficacy.

PW	LF	RV	LV	PB	FF	NS	ZO
	NB	PB	PB	PB	NM	NM	PB
	PM	NB	NM	PS	PS	PM	PS
	NM	NM	PS	NM	NM	NM	PS
	ZO	ZO	ZO	ZO	NM	NM	NB
	NB	NM	PS	PS	PS	NM	NM
	PS	NB	NM	ZO	NM	PS	PS
	PM	PM	PM	PS	NB	PS	NM
	FF	FF	FF	FF	FF	NB	NM
	FF	FF	FF	FF	FF	FF	FF

## Data Availability

The data used to support the findings of this study are available from the corresponding author upon request.

## Appendix

### A. The Synthesis Process of Force and Torque

(37)
$$\begin{array}{c} F_{5T}=c_{T}\left[-F_{5d}+F_{5p}\cos\theta_{3}+F_{5s}\cos\left(\theta_{3}+\sigma_{5}\right)-F_{5u}\cos\left(\theta_{3}+\sigma_{5}-\sigma_{u}\right)-F_{5m}\cos\left(\theta_{3}+\sigma_{5}+\sigma_{mo}\right)\right],\\ F_{5Y}=-F_{5p}\sin\left(\theta_{3}\right)+F_{5s}\sin\left(\theta_{3}+\sigma_{5}\right)-F_{5u}\sin\left(\theta_{3}+\sigma_{5}-\sigma_{u}\right)-F_{5m}\sin\left(\theta_{3}+\sigma_{5}+\sigma_{mo}\right),\\ M_{5Y}=0.5\left(L_{2}+L_{3}\right)F_{5Y}\cos\theta_{3},\\ M_{5T}=0.5\left(L_{2}+L_{3}\right)F_{5T}\sin\theta_{3},\\ F_{4T}=c_{T}\left(-F_{4s}+F_{4d}+F_{4p}\cos\theta_{2}+F_{4s}\cos\left(\theta_{2}+\sigma_{4}-\sigma_{u}\right)-F_{4m}\cos\left(\theta_{2}+\sigma_{4}+\sigma_{mo}\right)-F_{5f}\sin\theta_{3}\right),\\ M_{4T}=0.5L_{2}F_{4T}\sin\left(\theta_{2}\right),\\ F_{4Y}=-F_{4p}\sin\left(\theta_{2}\right)+F_{5s}\sin\left(\theta_{2}+\sigma_{4}\right)-F_{5u}\sin\left(\theta_{2}+\sigma_{4}-\sigma_{u}\right)-F_{5m}\sin\left(\theta_{2}+\sigma_{4}+\sigma_{mo}\right),\\ M_{4Y}=0.5L_{2}F_{4Y}\cos\left(\theta_{2}\right),\\ \left[\begin{array}{c} F_{4g}^{*}\\ M_{4g}^{*} \end{array}\right]=-I_{4}\left[\begin{array}{c} a_{4}\\ a_{d} \end{array}\right]+I_{4}\left[\begin{array}{c} \omega_{4}\times \upsilon_{4}\\ \omega_{4}\times \omega_{4} \end{array}\right],\\ F_{pg}^{2}=F_{5g}^{2}+F_{4g}^{2},\\ M_{pg}^{2}=M_{5g}^{2}+M_{4g}^{2}+M_{5f}^{2},\\ F_{Pz}^{2}=F_{4T}^{2}+F_{4Y}^{2}+F_{5T}^{2}+F_{5Y}^{2},\\ M_{pz}^{2}=M_{4T}^{2}+M_{4Y}^{2}+M_{5T}^{2}+M_{5Y}^{2}. \end{array}$$

### B. The Glossary (Namely, the Symbol Table)

*L*_*i*_: The length of the *i* joint as shown in Figure 3
*θ*_*i*_: The angle between the *i* joint and the horizontal surface as shown in Figures 4–6
*Ф*_*i*_: The angle between the *i* joint and the former joint as shown in Figures 3, 4, and 6
*t*: The time function, see Section 2.1.1, and as shown in Equation (35)
*μ*: Viscosity coefficient, see Section 2.1.1
Re: Reynolds number, see Section 2.1.1
*M*: Torque, see Section 2.1.1
*F*: Force, see Section 2.1.1
*I*: Inertial rotation inertia, see Section 2.1.1
*A*: Area, as shown in Equations (6)–(10)
*δ*: Angle of attack, as shown in Figure 4
*ρ*: Density, as shown in Equations (6)–(10)
Θ: The surface temperature of the robot dolphin, see Section 2.1.1
*c*_*i*_: Coefficient, see Section 2.1.1
*r*_*i*_^*j*^: The position vector, as shown in Equation (1)
*ω*: Angle speed, as shown in Equations (2)–(5)
*υ*: Linear speed, as shown in Equations (3) and (5)
*α*: Angular acceleration, as shown in Equation (4)
*a*: Line speed, as shown in Equation (5)
*s*: Sliding surface function, as shown in Equation (30), see Section 5.3.1
*e*: Error, as shown in Equation (30), see Section 5.3.1
*v*: Lyapunov function, as shown in Equation (33), see Section 5.3.1
*σ*_*s*_: Bounded positive variables, as shown in Equation (34), see Section 5.3.1
*U*_*t*_: Space speed vector of the robot dolphin, as shown in Equation (29), see Section 5.3.1
*x*: *x* direction vector, as shown in Equation (35), see Section 5.3.2
*y*: *y* direction vector, as shown in Equation (35), see Section 5.3.2.

## References

[1] Tong B. G., Zhuang L. X., Cheng J. Y. (1993). The hydrodynamic analysis of fish propulsion performance and its morphological adaptation. *Sadhana*.

[2] Scaradozzi D., Palmieri G., Costa D., Pinelli A. (2017). BCF swimming locomotion for autonomous underwater robots: a review and a novel solution to improve control and efficiency. *Ocean Engineering*.

[3] Chen X., Wu Z., Zhou C., Yu J. (2017). Design and implementation of a magnetically actuated miniature robotic fish∗. *IFAC-PapersOnLine*.

[4] Nguyen P. L., Lee B. R., Ahn K. K. (2016). Thrust and swimming speed analysis of fish robot with non-uniform flexible tail. *Journal of Bionic Engineering*.

[5] Liu J., Hu H. (2010). Biological inspiration: from carangiform fish to multi-joint robotic fish. *Journal of Bionic Engineering*.

[6] Wang J., Tan X. (2013). A dynamic model for tail-actuated robotic fish with drag coefficient adaptation. *Mechatronics*.

[7] Wang Y., Tan J., Zhao D. (2015). Design and experiment on a biomimetic robotic fish inspired by freshwater stingray. *Journal of Bionic Engineering*.

[8] Vo T. Q., Kim H. S., Lee B. R. (2009). Propulsive velocity optimization of 3-joint fish robot using genetic-hill climbing algorithm. *Journal of Bionic Engineering*.

[9] Wang M., Dong H., Li X., Zhang Y., Yu J. (2019). Control and optimization of a bionic robotic fish through a combination of CPG model and PSO. *Neurocomputing*.

[10] Ren G., Dai Y., Cao Z., Shen F. (2015). Research on the implementation of average speed for a bionic robotic dolphin. *Robotics and Autonomous Systems*.

[11] Ding R., Yu J., Yang Q., Tan M., Zhang J. (2011). Dolphin-like swimming modeling for a biomimetic amphibious robot. *World Congress*.

[12] Yu J., Liu J., Wu Z., Fang H. (2018). Depth control of a bioinspired robotic dolphin based on sliding mode fuzzy control method. *IEEE Transactions on Industrial Electronics*.

[13] Wu Z., Yang X., Zhou C., Yuan J., Yu J. Dynamics modeling and simulation for a gliding robotic dolphin.

[14] Wu Z., Yu J., Yuan J., Tan M., Qi S. (2020). Gliding motion regulation of a robotic dolphin based on a controllable fluke. *IEEE Transactions on Industrial Electronics*.

[15] Yuan J., Wu Z., Yu J., Tan M. (2017). Sliding mode observer based heading control for a gliding robotic dolphin. *IEEE Transactions on Industrial Electronics*.

[16] Suebsaiprom P., Lin C. L., Engkaninan A. (2017). Undulatory locomotion and effective propulsion for fish-inspired robot. *Control Engineering Practice*.

[17] Ren Q., Xu J., Fan L., Niu X. (2013). A GIM-based biomimetic learning approach for motion generation of a multi-joint robotic fish. *Journal of Bionic Engineering*.

[18] Bal C., Ozmen Koca G., Korkmaz D., Akpolat Z. H., Ay M. (2019). CPG-based autonomous swimming control for multi-tasks of a biomimetic robotic fish. *Control Engineering Practice*.

[19] Yang Y., Wang J., Wu Z., Yu J. (2018). Fault-tolerant control of a CPG-governed robotic fish. *Engineering*.

[20] Ren Q., Xu J., Li X. (2015). A data-driven motion control approach for a robotic fish. *Journal of Bionic Engineering*.

[21] Suebsaiprom P., Lin C. (2015). Maneuverability modeling and trajectory tracking for fish robot. *Control Engineering Practice*.

[22] Wu Z., Yu J., Tan M., Zhang J. (2014). Kinematic comparison of forward and backward swimming and maneuvering in a self-propelled sub-carangiform robotic fish. *Journal of Bionic Engineering*.

[23] Wu Z., Yu J., Su Z., Tan M. Implementing 3-D high maneuvers with a novel biomimetic robotic fish.

[24] Xie F., Zhong Y., du R., Li Z. (2019). Central pattern generator (CPG) control of a biomimetic robot fish for multimodal swimming. *Journal of Bionic Engineering*.

[25] Govardhan D., Ramulub P. J., Prasad R., Anbusagar N. R. R. (2018). Hydrodynamics of a fish useing fluid structure interaction. *Materialstoday: Proceedings*.

[26] Lin Z. W., Hess A., Yu Z., Cai S., Gao T. (2019). A fluid-structure interaction study of soft robotic swimmer using a fictitious domain/active-strain method. *Journal of Computational Physics*.

[27] Khalid M. S. U., Akhtar I., Imtiaz H., Dong H., Wu B. (2018). On the hydrodynamics and nonlinear interaction between fish in tandem configuration. *Ocean Engineering*.

[28] Zhang P., Krasner E., Peterson S. D., Porfiri M. (2019). An information-theoretic study of fish swimming in the wake of a pitching airfoil. *Physica D: Nonlinear Phenomena*.

[29] Chung H., Cao S. X., Philen M., Beran P. S., Wang K. G. (2018). CFD-CSD coupled analysis of underwater propulsion using a biomimetic fin-and- joint system. *Computers and Fluids*.

[30] Ghaffari S. A., Viazzo S., Schneider K., Bontoux P. (2015). Simulation of forced deformable bodies interacting with two-dimensional incompressible flows: application to fish-like swimming. *International Journal of Heat and Fluid Flow*.

[31] Zhou H., Hu T. J., Low K. H. (2015). Bio-inspired flow sensing and prediction for fish-like undulating locomotion: a CFD-aided approach. *Journal of Bionic Engineering*.

[32] Li K., Yu J., Wu Z., Tan M. Hydrodynamic analysis of a gliding robotic dolphin based on computational fluid dynamics.

[33] Tang M.-F., Xu T. J., Dong G.-H., Zhao Y.-P., Guo W.-J. (2017). Numerical simulation of the effects of fish behavior on flow dynamics around net cage. *Applied Ocean research*.

[34] Bergmann M., Iollo A. (2011). Modeling and simulation of fish-like swimming. *Journal of Computational Physics*.

[35] Xia D., Chen W. S., Liu J. K., Wu Z. (2016). Effect of head swing motion on hydrodynamic performance of fishlike robot propulsion. *Journal of Hydrodynamics*.

[36] He W., Wang T., He X., Yang L.-J., Kaynak O. (2020). Dynamical modeling and boundary vibration control of a rigid-flexible wing system. *IEEE/ASME Transactions on Mechatronics*.

[37] Virgala I., Kelemen M., Božek P. (2020). Investigation of snake robot locomotion possibilities in a pipe. *Symmetry*.

[38] Chopra M. G. (1974). Hydromechanics of lunate-tail swimming propulsion. *Journal of Fluid Mechanics*.

[39] Fish F. E., Hui C. A. (1991). Dolphin swimming-a review. *Mammal Review*.

[40] Su Z., Yu J., Tan M., Zhang J. (2014). Implementing flexible and fast turning maneuvers of a multijoint robotic fish. *IEEE/ASME Transactions on Mechatronics*.

[41] Pham V. A., Nguyen T. T., Vo T. Q. Turning motion direction of fish robot driven by non-uniform flexible pectoral fins.

[42] Zonggang L. I., Weijun M. A., Liming G. E., Yajiang D. U. (2016). Research on turning characteristics of a biomimetic robotic boxfish driven by pectoral fin with two degrees of freedom. *Roboctic*.

[43] Weihs D. A. (1972). Hydrodynamical analysis of fish turning manoeuvres. *Proceedings of the Royal Society B: Biological Sciences*.

[44] Liu J., Wu Z., Yu J., Cao Z. Flippers-based turning analysis and implementation of a dolphin robot.

[45] Yu J., Li Y. F., Wang M., Tan M. Turning analysis and its implementation of link-based dolphin-like robots.

[46] Chen J. W., Zhu H., Zhang L., Sun Y. (2018). Research on fuzzy control of path tracking for underwater vehicle based on genetic algorithm optimization. *Ocean Engineering*.

[47] Yang Z., Wan L., Sun X., Chen L., Chen Z. (2016). Sliding mode control for bearingless induction motor based on a novel load torque observer. *Journal of Sensors*.

[48] Wang R., Cheng L., Tan M. (2019). Prediction-based seabed terrain following control for an underwater vehicle manipulatorsystem. *IEEE Transactions on Systems, Man, and Cybernetics: Systems*.

[49] Kelasidi E., Pettersen K. Y., Kohl A. M., Gravdahl J. T. (2017). An experimental investigation of path following for an underwater snake robot with a caudal fin ∗. *IFAC-Papers OnLine*.

[50] Qingzheng X., Wang Z., Zhen Z. (2020). Information fusion estimation-based path following control of quadrotor UAVs subjected to Gaussian random disturbance. *ISA Transactions*.

[51] Li Z., Chen L., Zheng Q., Dou X., Yang L. (2019). Control of a path following caterpillar robot based on a sliding mode variable structure algorithm. *Biosystemsengineering*.

[52] Das P. K., Behera H. S., Panigrahi B. K. (2016). Intelligent-based multi-robot path planning inspired by improved classical Q-learning and improved particle swarm optimization with perturbed velocity. *Engineering Science and Technology, an International Journal*.

[53] Ma H., Li Y. (2020). A novel dead zone reaching law of discrete-time sliding mode control with disturbance compensation. *IEEE Transactions on Industrial Electronics*.

[54] Ma H., Li Y. (2019). A generalized input-output-based digital sliding-mode control for piezoelectric actuators with non-minimum phase property. *International Journal of Control, Automation and Systems*.

[55] Xue Z., Liu J., Wu Z., du S., Kong S., Yu J. (2019). Development and path planning of a novel unmanned surface vehicle system and its application to exploitation of Qarhan Salt Lake. *Science China (Information Sciences)*.

[56] Bozek P., Karavaev Y. L., Ardentov A. A., Yefremov K. S. (2020). Neural network control of a wheeled mobile robot based on optimal trajectories. *International Journal of Advanced Robotic Systems*.

[57] He W., Mu X., Zhang L., Zou Y. (2021). Modeling and trajectory tracking control for flapping-wing micro aerial vehicles. *IEEE/CAA Journal of Automatica Sinica*.

